# The Lewis Histo-Blood Group System: Molecular Analysis of the 59T>G, 508G>A, and 1067T>A Polymorphisms in an Amazonian Population

**DOI:** 10.1371/journal.pone.0069908

**Published:** 2013-07-29

**Authors:** Tereza Cristina de Oliveira Corvelo, Rosane do Socorro Pompeu de Loiola, Délia Cristina Figueira Aguiar, Gyselly de Cássia Bastos de Matos, Danielle Calado de Brito

**Affiliations:** 1 Immunogenetics Laboratory, Biological Sciences Institute, Federal University of Pará, Belém, Pará, Brazil; 2 Central Laboratory Pará State, Executive Office of Health Pará State, Belém, Pará, Brazil; Institut Jacques Monod, France

## Abstract

**Background:**

The Lewis (*FUT3*) gene is responsible for the expression of the Le^a^ and Le^b^ blood group antigens. The individuals, who not synthesize these antigens have the phenotype Lewis negative, due to the presence of some single nucleotide polymorphisms (SNPs), such as 59T>G, 508G>A and 1067T>A, whose distribution is different in various ethnic groups. Our aim was to verify the frequencies of these SNPs in an admixed population of Belém-Pará-Brazil.

**Materials and Methods:**

Polymerase chain reaction/restriction enzyme method were used to detect these SNPs in the *FUT3* gene, whereas Lewis phenotypes were defined by the direct hemagglutination and in saliva by Dot-Elisa assay in a random sample of 150 individuals from admixed population of Belém in the northeast Brazilian Amazon region.

**Results:**

The frequency of these SNPs was detected as 47.6% (59T>G), 17.3% (508G>A) and 5.3% (1067T>A).The discrepancies between blood and salivary Lewis phenotypes are related to the relatively high frequencies of 59T>G and the null allele 508G>A. Whereas 38.6% of the individuals were Lewis negative based on blood, only 17.24% also tested negative when their saliva were analyzed.

**Conclusion:**

We have found a marked consistency between the phenotypes and genotypes of the Lewis blood group system. Furthermore, our obtained F_ST_ values reveal distinct frequencies of the *FUT3* SNPs between the present sample and its representative ancestral populations. These observations will help to evaluate the Lewis antigens impact as susceptibility markers, in genetic association studies to certain diseases.

## Introduction

The Lewis antigens were discovered in the erythrocytes, although they are synthesized in the epithelium and then incorporated through the membrane of the erythrocytes from the plasma [1]–[6].

The Lewis antigens are biochemically related to the ABH antigens, being produced from the same precursor substances. The Lewis^a^ and Lewis^b^ are the principal antigens of this system [7]. Given this, the Lewis blood group presents a number of different phenotype classes – the Le(a+b-) type, which is the non-secretor phenotype, the Le(a+b+) or weak secretor (Sew), which increases the availability of the type I precursor for modification into the Le^a^ antigen and a reduction in salivary ABH substances. The Le(a−b+) phenotype, which is found in individuals with the Se gene, results from the association between the Le^a^ specificity and the Le^d^ (type H-1) antigen determinant, resulting in the Le^b^ type antigen, a product of the epistatic interaction between the secretor and Lewis loci [8]. Finally, the Le(a−b−) phenotype involves a number of different alleles of the Lewis (*Le*) gene which codify non-functional transferases, and are labeled *le*. In this case, the individuals, whether secretors or not, do not express the Le^a^ or Le^b^ antigens.

The silent variant of the Lewis gene (*le*) contain single nucleotide polymorphism (SNP), many of which inactivate the enzyme [9]. The most common haplotype variations correspond to the *le^59/508^*, which have been detected in Asian (24%) and African (19%) populations, while the *le^202/314^* (17%) and *le^59/1067^* (4%) were found mainly in European populations [10]–[12]. The 508G>A, and 1067T>A SNPs, which are both found in the catalytic domain of the enzyme, inactivate the product of the Lewis gene, while the 59T>G SNP, in the trans-membranous domain of this protein, only reduces its enzymatic activity rather than eliminating it altogether [9].

The frequency of the different Lewis phenotypes varies significantly among different ethnic groups. The Le(a-b+) phenotype is the most common overall, but varies from 75% in Europeans to 61% in Africans, and 42% in Asians [13], [14], while the Le(a−b−) phenotype is more frequent in Africans (19%), with more than double the frequency recorded in Europeans (8%) and Asians (7%).

Some individuals present changes in the expression of the Lewis antigens (which may be absent altogether) when affected by certain diseases and/or physiological conditions, especially in the erythrocytes, due to their secondary acquisition by these cells. In this case, some individuals that are Le(a−b−) in their blood present Le^b^ in their secretions [15]–[17]. Given this, Ørntoft *et al.,* [18] classified Le(a−b−) individuals in two distinct groups: the “genuine” group, in which antigens are not found in the blood or the saliva, and there is no enzymatic activity, and the “non-genuine” group, in which there are no antigens in the blood, but they are expressed in the saliva, together with activity of the Lewis FUT3 enzyme.

Understanding the complexity of the polymorphisms of the Lewis system is especially important for defining the function of these antigens as markers for the differentiation of the normal condition and pathological alterations observed in human tissue. As the expression of the Lewis antigens in the blood does not always allow the identification of the true phenotype, the present study investigated the frequency of the 59T>G, 508G>A, and 1067T>A SNPs, and their effects on the expression of the phenotypes of these antigens in the population of Belém a city of Pará state in the northern Brazil.

## Materials and Methods

### Sample

This study analyzed samples of blood and saliva from 150 unrelated and randomly-selected individuals (89 women and 61 men, with a mean age of 34.6±14.5 years) from the admixed population of Belém in the northeast Brazilian Amazon region. The major groups involving in the admixture process of the Belém population were mainly Portuguese (47%), Africans (23%) and Native Indians (30%). These estimated proportions of ethnic admixture are based on a previous study of Guerreiro *et al.,* [19], using as marker the ABO system.

In the attempt to control the population heterogeneity and for operational convenience, the sample collection is randomly stratified by the 8 administrative districts that comprise the city of Belém. According to the proportion of the population of each district the individuals have been randomly-selected from the spontaneous demand in the Central Laboratory, which is reference laboratory for clinical analysis in the state of Pará.

The study was approved by the Ethics in Research Committee of the Tropical Medicine Nucleus of the Federal University of Pará, and all the study subjects agreed in writing to participate in the study after reading an informed consent form.

### Blood Phenotypes and ABH and Lewis Secretor Status

A 5 ml sample of peripheral blood was obtained from each participant and stored in a tube containing heparin. The phenotypes of the ABO and Lewis systems were determined by the conventional direct hemagglutination technique, using the monoclonal anti-A, anti-B, anti-H, anti-Le^a^, and anti-Le^b^ antibodies (Fresenius Hemocare Brasil Ltda).

The ABH and Lewis secretor status of the subjects was determined by DOT-ELISA assay, based on the technique described by Pflug *et al.,* [20], using the monoclonal anti-A (1∶100), anti-B(1∶50), anti-H (1∶50), anti-Le^a^ (1∶500), and anti-Le^b^(1∶1000) antibodies from Fresenius Hemocare Brazil.

### Amplification of the *FUT3* Gene by Polymerase Chain Reaction (RFLP-PCR)

The *FUT3* gene was genotyped for the identification of the 59T>G and 508G>A mutations using the sn3-sn4 and sn8-sn9 primers, respectively (Table 1). In order to detect the 59T>G SNP, the sense primer sn3 induces the production of an *Mspl* site in the amplified fragment of the mutant allele. The amplified product of the mutant allele was cleaved into two fragments of 68 and 25 base pairs (bps) by digestion with *Mspl*. To detect the 508G>A SNP, the sn8-sn9 primer set was used to amplify a fragment of 206 bps and induce a cleavage site for *PvuII*, which resulted in the production of two fragments, of 104 bps and 102 bps.

**Table 1:** Amplification conditions for the *FUT3* gene and its restriction sites for the different endonucleases analyzed in the present study.

Primer	Sequence (5′-3′)	°C annealing/time	Fragment size (bp)	Enzyme	Site
Sn3*	5′-CCATGGCGCCGCTGTCTGGCCGCCC-3′	62°/30 seconds	93	MspI	5′-C↓C G G-3′
Sn4*	5′-AGTGGCATCGTCTCGGGACACACG-3′				
Sn8*	5′-ACTTGGAGCCACCCCCTAACTGCCA-3′	65°/45 seconds	206	Pvu II	5′-CAG↓CTG-3
Sn9*	5′-TGAGTCCGGCTTCCAGTTGGACACC-3′				
Sn6*	5′-CGCTCCTTCAGCTGGGCACTGGA –3′	67°/45 seconds	109	Hind III	5′-A↓AGCTT-3′
Sn7*	5′-CGGCCTCTCAGGTGAACCAAGAAGCT- 3				
P1**	5′-ATGATGGAGACGCTGTCCCGGTACAAGTT-3′	69°/1 minute	400		
	5′-CGGCCTCTCAGGTGAACCAAGAAGCT-3′				

* Kudo*et al.,* [21];

** Francez *et al.*; [22].

To detect the 1067T>A SNP, an initial amplification was conducted using the P1 primers (Table 1), which produced a fragment of 400 bps. Using the product of this first reaction as a template, a nested PCR was used to amplify an internal fragment of 109 bps, using the sn6–sn7 primers to create a site for *HindIII* in the mutant allele, generating fragments of 85 and 64 bps. The PCRs were based on 1 µL of genomic DNA, 5 pmol of each primer, 1.25 mM of dNTP, 2 mM of MgCl2, 0.5 unit of Taq polymerase in 2.5 µl of buffer (50 mM KCl, 10 mMTris-HCl, pH 8.3). A negative control (amplification with no DNA sample) was included in all runs. The products were analyzed by electrophoresis in 2% agar gel colored with ethidium bromide. Markers of standard DNA with molecular weights of 50 bps and 100 bps from Fermentas Life Science were used in all procedures.

### Statistical Analysis

The distribution of frequencies and proportions was processed using the Bioestat 5.0 program of Ayres *et al*. [23]. The ARLEQUIN package (version 3.1, 2006) was used to estimate haplotype frequencies and run the tests for Hardy-Weinberg equilibrium and linkage disequilibrium.

## Results

The analysis of the blood of the 150 subjects returned the following phenotype frequencies for the Lewis system: 57% (85/150) presented the Le(a−b+) phenotype and 4% (7/150) were Le(a+b+), while 39% (58/150) presented phenotype Le(a−b−). In the latter group, 82.76% (48/58) of the individuals expressed the Lewis antigens in the saliva, and were this classified as nongenuine Lewis-negative. The remaining 10 subjects presented no antigens in the saliva, and were classified as genuine Lewis-negative.

Three very common SNPs –59T>G, 508G>A, and 1067 T>A – were analyzed in the *FUT3* gene. Overall, seven different haplotypes were inferred for the 150 subjects, in which the alleles with the isolated *Le^59^* or *le^59/508^* SNP were the most common. By contrast, alleles with the isolated *le^508^* and *le^1067^* SNPs or the *le^59/1067^* and *le^59/508/1067^* combinations were the rarest. The genotype and haplotype frequencies observed for the Lewis gene (*FUT3*) are shown in Table 2.

**Table 2:** Allele and genotype frequencies for the *FUT3* loci analyzed in the sample from the population of Belém in the northeast Brazilian Amazon region.

*Locus*/genotype	Frequency		Allele	2n = 300	Frequency	±SD
	Absolute	Relative				
	n	%				
*Le Le*	23	15.33	*Le*	149	0.497	±0.029
*Le Le^59^*	62	41.33	*Le^59^*	87	0.290	±0.026
*Le le^59,1067^*	5	3.33	*le^59,508^*	46	0.153	±0.021
*Le le^59,508^*	28	18.66	*le^59,1067^*	6	0.020	±0.008
*Le le^1067^*	5	3.33	*le^508^*	2	0.007	±0.005
*Le le^59,508,1067^*	3	2.00	*le^1067^*	6	0.020	±0.007
*Le^59^ Le^59^*	11	7.33	*le^59,508,1067^*	4	0.013	±0.007
*Le^59^ le^59,508^*	3	2.00				
*le^59,508^ le^59,1067^*	1	0.67				
*le^59,508^ le^59,508^*	6	4.00				
*le^508^ le^508^*	1	0.67				
*le^59,508^ le^59,508,1067^*	1	0.67				
*le^59,508^ le^1067^*	1	0.67				

The 59T>G polymorphism had an overall frequency of 47.66%, being detected in 121 individuals, of which, 22 were homozygous and 99 heterozygous. The 508G>A SNP was much rarer, with a frequency of 17.33%, being detected in 44 individuals, of which eight were homozygous, included one sample which presented the isolated 508G>A SNP. The 1067T>A SNP was found only in the heterozygous form, at a frequency of 5.3%, with the isolated from being recorded in six individuals, and the combined form, with *Le^59^* or *le^59/508^* SNP, in six and four cases, respectively. The distribution of the Lewis genotypes according to the ABO and Lewis blood group phenotypes are presented in table 3.

**Table 3:** Lewis and ABO blood group phenotypes and *FUT3* genotypes recorded for the individuals from Belém in the northeast Brazilian Amazon region.

Lewis/ABO blood phenotype		Lewis Genotype					Total	%
		*LeLe*	*LeLe^59^*	Lele*	*Le^59^Le^59^*	le*le*		
Positive Lewis	O	13	32	12			57	38,0
	A	7	9	7			23	15,3
	B	3	4	4			11	7,3
	AB	0	1	0			1	0,7
Negative Lewis								
Genuine	O					6	6	4,0
	A					2	2	1,3
	B					2	2	1,3
	AB					0	0	
Non-Genuine	O		7	10	5		22	14,7
	A		6	10	5		21	14,0
	B		1	0	3		4	2,7
	AB		0	0	1		1	0,7
**Total**		**23**	**60**	**43**	**14**	**10**	**150**	**100**

le*: 59/508 and/or 59/1067.

The rates of heterozygosity recorded for the SNPs at positions 59T>G, 508G>A, and 1067T>A were 66%, 24%, and 11%, respectively. Analysis of the *FUT3* genotype frequencies indicated that the study population was not in Hardy-Weinberg equilibrium (p<0,01). The analysis of linkage disequilibrium between the pairs of combined sites also indicated a highly significant deviation (χ^2^ = 26.94, d.f. = 1, p<0.0001) between the combinations of alleles at sites 59 T>G and 508 G>A.

Given the considerable complexity of the polymorphisms of the Lewis (*FUT3*) gene, the different genotypic and phenotypic configurations were grouped in the following categories (see Table 3):

- Positive Lewis - included 92 individuals with the positive Lewis blood group phenotype, who were secretors of ABH, Le^a^ and Le^b^ antigens;
- Genuine Lewis-negative (phenotypically Le(a−b−) in blood and saliva) –10 individuals with the genuine Le(a−b−) blood phenotype, which all presented the *le^59/508^* and/or *le^59/1067^* haplotypes in the homozygous condition. Among these individuals 2 were ABH and Lewis non-secretors and 8 were only ABH secretors.
- Non-genuine Lewis-negative (characterized by Le(a−b−) in blood but with expression of the Le^a^ and/or Le^b^ antigens in saliva) – included 48 individuals that had the 59T>G SNP in homozygote (n = 14) or heterozygote (n = 14). In some cases (n = 20), this SNP was combined with the 508G>A and/or 1067T>A null alleles in the heterozygous condition. In this group, 10 individuals secreted only the Le^a^ substance in saliva, so that they were ABH non-secretors, while 38 individuals were ABH and Lewis secretors.

Of the Lewis-positive individuals, 75% (69/92) presented heterozygous genotypes (Le/_), while the other 25% were homozygous for the Le allele (Le/Le). In the case of the non-genuine Lewis-negative individuals, 70.83% (34/48) were heterozygous (Le/−) and 29.17% (14/48) were homozygous for the 59T>G SNP (*Le^59^*/*Le^59^*). Then, the proportion of individuals which are heterozygous for the *le^59/508^* and/or *le^59/1067^* haplotypes is significantly higher for the non-genuine Lewis-negative individuals (41.7% vs. 25%; p = 0.034 for Fisher’s exact test). On the other hand, the proportion of individuals that are heterozygous for the isolated 59 T>G SNP is significantly higher in the group with the Lewis-positive phenotype (50,0% vs 29.16%; p = 0.0138 for Fisher’s test).

In the heterozygous individuals the number of inactive (le*) alleles in the group non-genuine Lewis-negative phenotype is approximately double that found in those with the Lewis-positive phenotype, with the opposite pattern being observed for the mutant *Le^59^* allele.

On the other hand, in the non-genuine Lewis-negative individuals, non-O blood group phenotypes (in particular A1) were most common, with 54.17% (26/48) of the cases, whereas in the Lewis-positive individuals, non-O phenotypes were present in 38.04% (35/92) of the individuals (p = 0.05 for Fisher’s test). All these differences between positive and non-genuine Lewis-negative individuals can be visualized and conferred in Figure 1.

**Figure 1:** Genotype frequencies for the Lewis (*FUT3*) gene and non-O blood groups in the positive and non-genuine Lewis-negative individuals.

Significantly different F_ST_ values (Table 4) were found comparing the *FUT3* allele frequencies with those available in the literature [11] for European, African, and Asian ethnic groups (Figure 2).

**Figure 2:** Comparison of the allele frequencies for the *FUT3* gene recorded in different populations. The frequencies for the African (Accra, Ghana), European (Caucasians from Coriell and Camden, NJ, USA), and Asian (Ulaanbaatar, Mongolia) were obtained from Soejima*et al.* [11]. Alleles not detected in the present study are designated by an asterisk (*).

**Table 4:** The F_ST_ values for pairwise comparisons of haplotype frequencies of the *FUT3* gene between the present study and other populations.

Population	1	2	3	4
Belém (1)	0.00000			
European (2)*	0.11172	0.00000		
African (3)*	0.09219	0.11934	0.00000	
Asian (4)*	0.07608	0.07691	0.06759	0.00000

* Soejima *et al*.; [11].

## Discussion

Traditionally, the expression of the Lewis antigens has been determined in relation to erythrocyte levels, although as they are primarily histoantigens of the blood group, they can be detected more accurately in salivary secretions [1]–[3].

In the present study, 92 of the 150 study subjects had Lewis-positive phenotypes, which were identified by the presence of at least one *Le* allele codifying an active Lewis enzyme. The other 58 subjects all presented the Lewis-negative phenotype, based on conventional hemagglutination. A result of the study was the fact that most of these cases (82.76%, 48/58) presented the Lewis antigen in their saliva, contradicting the negative result from the blood samples.

The molecular analyses of the *FUT3* gene resulted in the identification of three principal SNPs, at positions 59T>G, 508G>A, and 1067T>A, which are known to account for 90% of the Lewis-negative phenotypes in Europeans, confirming the presence of the corresponding genotype combination, as predicted by existing knowledge of the effects of the isolated SNPs or haplotypes. However, the haplotypes corresponding to the Lewis genotypes cannot be determined reliably in all cases.

Based on the available data [10, 21, 24–25], it can be inferred that the individuals with SNP 59T >G associated with 508G>A or 1067T>A have a cis type chromosomal distribution, given that trans-type arrangements are uncommon. In this context, an overview of the distribution of the mutations investigated in the present study indicates that, in addition to the functional Le allele, there are two predominant alleles in this group, one with the *Le^59^* SNP, and the other with SNPs at positions 59T>G and 508G>A (*le^59/508^*). This distribution of alleles is effectively ambiguous, because heterozygous individuals that were either *Le/Le^59^* or *Le/le^59/508^* were recorded in both positive and negative Lewis blood groups. In addition, when null alleles, that is, *le^59/508^*, *le^59/1067^*, *le^1067^*, *le^508^*, and *le^59/508/1067^*, were homozygous, the individuals presented the genuine Lewis-negative phenotype, which determines the absence of the expression of Lewis antigens in both the blood and the saliva, confirming the inactivating effect of these SNPs located in the catalytic domain [10].

In the present study, the 59T>G SNP, either homo- or heterozygous and isolated or in combination with other null mutations, was recorded in all individuals with Lewis antigens in the saliva, but with negative results for the blood samples. Given this, the pattern of blood-saliva discrepancies in the characterization of the Lewis phenotypes is consistent with that observed in previous studies, in which the non-genuine Lewis-negative trait was related to the presence of this type of mutation in the trans-membranous region [9], [26]–[27].

In addition, studies in enzymatic kinetics have shown that the enzyme produced by the *Le^59^* allele does not act on the glycolipids, due to its differentiated activity in relation to the acceptor substrates, that is, glycolipids versus glycoproteins [28], which results in an absence of specific Le^a^ and Le^b^ factors in the plasma and, thus, an Le(a−b−) blood phenotype. Experimental molecular studies have shown that the isolated 59T>G SNP presents a reduction of approximately 50% in the levels of the FUT3 enzyme, which is probably a result of the reduction in its potential for retention in the Golgi complex, although it is normally present in conjunction with the 508G>A and 1067T>A SNPs [9]–[10], [29]. These SNPs at sites 508G>A and 1067T>A, in turn, reduce fucosyltransferase activity either completely or to levels below 10% of normal [10].

One other aspect that has been analyzed in previous studies is the correlation between the amount of Lewis enzyme and the level of expression of the Le^a^ antigens in the intestinal mucosa, in particular, that the quantity of Le^a^ in the samples of Le/Le individuals was approximately twice that of the Le/le heterozygotes, indicating a regulatory effect of the Lewis gene [29]. This pattern could be observed in the non-genuine Lewis-negative individuals, especially in the case of the 59T>G SNP, which was well-represented in this group, with the levels of Le^a^ antigens in the saliva varying considerably, but randomly between the heterozygotes and homozygotes, invariably being reduced.

It seems likely that a set of genetic and epigenetic factors interact to limit the activity of the FUT3 enzyme, which may then synthesize quantities of antigens that are undetectable in serological tests, resulting in the apparent expression of the Lewis-negative phenotype. In addition, this data also provides the different proportions between the inactive alleles, which compose the heterozygote frequencies of Lewis-positive and non-genuine Lewis-negative individuals, illustrating the known genetic dosage effect, which has been demonstrated in a previous study by Nishihara *et al.,* [29].

One interesting result of the present study was the predominance of non-O blood groups in non-genuine Lewis-negative individuals. This may be explained by the fact that the biosynthetic routes of the ABH and Lewis antigens are related, and cause competition between the A/B glycosyltransferases and the Lewis fucosyltransferases for the common type 1 H precursor. This leads to a reduction in the number of Le^b^ epitopes in comparison with group O individuals, which can interfere with the power of recognition of some Lewis antibodies, resulting in positive individuals which are characterized as being negative [30].

Given this, individuals that have the heterozygous *FUT3* genotype and/or blood group A1 are the most likely to express the non-genuine Lewis-negative phenotype, indicating that the negatively modulating effect of the 59T>G SNP may be accentuated under certain circumstances, either pathological (e.g., inflammations, cancer or metabolic diseases) or physiological conditions, such as pregnancy, which may cause a reduction in the circulatory concentration of active Lewis glycolipids, resulting in the incompatible expression of Lewis antigens in the blood [15], [31]–[32].

According to the distribution of frequencies recorded in previous studies [9]–[10], [24], the 59T>G SNP is normally present in conjunction with the 508G>A and 1067T>A SNPs of the *FUT3* gene. In the present study, by contrast, the isolated form of the *Le^59^* allele was present at a relatively high frequency, which indicates the possibility that other combinations of 59T>G may exist, involving mutations that were not investigated in this population. An even more likely explanation may be the ethnic composition of the sample and the dynamics of the population, considering the possible contribution of its Amerindian component to the frequency of the *Le^59^* allele, although this group has not been studied in detail. The differences in the frequencies of the *FUT3* SNPs observed between the present sample and its representative ancestral populations (Table 4) may be the result of the admixture process, given that the population of Belém city is highly distinct, in genetic terms, from the populations from which it is derived [19].

Overall, the results of the present study indicated a marked consistency between the phenotypes and genotypes of the Lewis blood group system. The molecular analyses conducted in the present study helped to elucidate the serological discrepancies in phenotypes through the identification of the different mutant alleles and their respective frequencies, especially those related to the individuals classified as non-genuine Lewis-negative. In addition, our obtained F_ST_ values reflect the distinct frequencies of the FUT3 SNPs between Belém and its ancestral populations [11]. These findings will require further, more detailed investigation in order to provide a more definitive understanding of the function of these antigens as markers for the differentiation of normal and pathological conditions, and their involvement in immune and inflammatory responses of the organism which may affect the susceptibility and resistance of the individual to specific diseases.
